This article has been retracted.

# Identification and Validation of Key Genes in Hepatocellular Carcinoma by Bioinformatics Analysis

**DOI:** 10.1155/2021/6662114

**Published:** 2021-02-23

**Authors:** Jia Wang, Rui Peng, Zheng Zhang, Yixi Zhang, Yuke Dai, Yan Sun

**Affiliations:** ^1^Department of Molecular Medicine and Cancer Research Center, Chongqing Medical University, Chongqing, China; ^2^Department of Bioinformatics, Chongqing Medical University, Chongqing, China

## Abstract

Hepatocellular carcinoma (HCC) is the most frequent primary liver cancer and has poor outcomes. However, the potential molecular biological process underpinning the occurrence and development of HCC is still largely unknown. The purpose of this study was to identify the core genes related to HCC and explore their potential molecular events using bioinformatics methods. HCC-related expression profiles GSE25097 and GSE84005 were selected from the Gene Expression Omnibus (GEO) database, and the differentially expressed genes (DEGs) between 306 HCC tissues and 281 corresponding noncancerous tissues were identified using GEO2R online tools. The protein-protein interaction network (PPIN) was constructed and visualized using the STRING database. Gene Ontology (GO) and KEGG pathway enrichment analyses of the DEGs were carried out using DAVID 6.8 and KOBAS 3.0. Additionally, module analysis and centrality parameter analysis were performed by Cytoscape. The expression differences of key genes in normal hepatocyte cells and HCC cells were verified by quantitative real-time fluorescence polymerase chain reaction (qRT-PCR). Additionally, survival analysis of key genes was performed by GEPIA. Our results showed that a total of 291 DEGs were identified including 99 upregulated genes and 192 downregulated genes. Our results showed that the PPIN of HCC was made up of 287 nodes and 2527 edges. GO analysis showed that these genes were mainly enriched in the molecular function of protein binding. Additionally, KEGG pathway analysis also revealed that DEGs were mainly involved in the metabolic, cell cycle, and chemical carcinogenesis pathways. Interestingly, a significant module with high centrality features including 10 key genes was found. Among these, CDK1, NDC80, HMMR, CDKN3, and PTTG1, which were only upregulated in HCC patients, have attracted much attention. Furthermore, qRT-PCR also confirmed the upregulation of these five key genes in the normal human hepatocyte cell line (HL-7702) and HCC cell lines (SMMC-7721, MHCC-97L, and MHCC-97H); patients with upregulated expression of these five key genes had significantly poorer survival and prognosis. CDK1, NDC80, HMMR, CDKN3, and PTTG1 can be used as molecular markers for HCC. This finding provides potential strategies for clinical diagnosis, accurate treatment, and prognosis analysis of liver cancer.

## 1. Introduction

Liver cancer is the sixth most prevalent cancer and ranks second in terms of tumor-related mortality worldwide. Over half the new cases and deaths occur in China [1]. Primary liver cancer comprises hepatocellular carcinoma (HCC), intrahepatic cholangiocarcinoma (iCCA), and other rare tumors, notably fibrolamellar carcinoma and hepatoblastoma. Globally, HCC accounts for 90% of all cases of primary liver cancers and may arise in conjunction with one or more risk factors [2]. HCC is also characterized by high complexity, difficulty of early diagnosis, and easy recurrence, metastasis, and heterogeneity after surgical resection [3]. The overall prognosis of patients with HCC remains dismal [4]. Recently, many studies have shown that multiple genes and cellular pathways participate in the occurrence and development of HCC. However, the exact mechanisms are still largely unknown.

The development of large-scale parallel technologies, such as microarrays and sequencing, has rapidly reduced the cost of obtaining high-throughput data [5] and promoted the construction of large tumor databases such as The Cancer Genome Atlas (TCGA) [6]. In recent years, bioinformatics analysis of microarray technology and rapid processing of massive datasets have enabled the comprehensive identification of hundreds of differentially expressed genes (DEGs) involved in the occurrence and development of liver cancer [7]. Bioinformatics methods have been extensively employed to explore the underlying molecular mechanisms of HCC development and to reveal the key genes and pathways involved [8–10]. Through bioinformatics analysis and processing, a series of changes can be observed from a more accurate perspective, thereby identifying key biomarkers as targets for clinical drug trials [11]. This approach provides a new way to understand the molecular mechanisms underpinning the occurrence and development of HCC. Additionally, it has promise in accelerating the early detection, diagnosis, and treatment of HCC [12, 13].

The goals of this study were to construct an HCC-related protein-protein interaction (PPI) network and to identify the core genes using bioinformatics methods. Microarray datasets were downloaded from the Gene Expression Omnibus (GEO) database, and the DEGs between HCC tissues and corresponding noncancerous tissues were identified. Functional enrichment was analyzed using DAVID 6.8 [14], and modules were also detected in the PPIN using Cytoscape. The genes with high centrality features were considered the potential critical genes and included in the first-ranked module. Additionally, three frequently used centralities were calculated for each protein in the HCC-related PPIN: degree centrality, betweenness centrality, and closeness centrality [15]. Furthermore, five HCC-related key genes were identified by cBioPortal. The results were verified by quantitative real-time fluorescence polymerase chain reaction (qRT-PCR) in a normal human hepatocyte cell line (HL-7702) and three HCC cell lines (SMMC-7721, MHCC-97L, and MHCC-97H). The survival of patients with upregulated expression of these five key genes was significantly worse. This study has furthered understanding of the development of HCC at the molecular level and identified potential molecular targets for new intervention strategies.

## 2. Materials and Methods

### 2.1. Microarray Data

The gene expression profiles GSE84005 and GSE25097 were obtained from the Gene Expression Omnibus database (http://www.ncbi.nlm.nih.gov/geo/). The GSE84005 [16] dataset included mRNA and lncRNA gene expression profile data of 38 HCC tissue samples and 38 adjacent nontumor samples. GSE25097 [16, 17] consisted of transcriptome profiling of 268 HCC tumor samples, 243 adjacent nontumor samples, 40 cirrhotic samples, and six healthy liver samples. The mRNA expression profiles of the 38 HCC tissue samples and 38 adjacent nontumor samples from GSE84005 and 268 HCC samples and 243 adjacent nontumor samples from GSE25097 were selected for follow-up studies.

### 2.2. Data Preprocessing and DEG Screening

GEO2R (http://www.ncbi.nlm.nih.gov/geo/geo2r/) [18], an online tool based on R language, was used to calculate the DEGs between the HCC and adjacent nontumor samples. It can analyze microarray data by using limma to provide multiple testing corrections. The Benjamini-Hochberg false discovery rate was selected to adjust for the occurrence of false-positive results. After data preprocessing, ∣logFC | >1.5, *q* < 0.01 was set. DEGs were selected for further study. Raw data from the Gene Expression Omnibus database was downloaded to unify the gene ID, and DAVID 6.8 (https://david.ncifcrf.gov/), an online analysis tool, was used to perform the gene ID conversion. Subsequently, the intersections of 99 upregulated genes and 192 downregulated genes from GSE25097 and GSE84005 were obtained using Venny 2.1. A total of 291 major DEGs were identified.

### 2.3. Construction of PPIN

STRING is a database of predicted or experimentally verified functional interactions among proteins [19]. Protein-protein interactions were downloaded from the STRING database version 10.0 (https://string-db.org/). A PPI network of DEGs was constructed, and a TSV file was generated by STRING, containing the full name and functional profile of each gene.

Cytoscape 3.7.0 (http://www.cytoscape.org/) is software capable of rapid and efficient biological analysis, which requires a download of the corresponding JAVA version to support its operation. The TSV file of the PPIN of DEGs was output from the STRING database and input into Cytoscape to construct a visual network of protein-protein interactions [20].

### 2.4. Gene Ontology and KEGG Pathway Enrichment Analyses

DAVID 6.8 (https://david.ncifcrf.gov/) is a database with annotation, visualization, and integrated discovery functions [14]. The annotation table is its main analysis tool, which contains functional annotation charts, functional annotation clustering, and functional annotation table subtools. Gene Ontology (GO) and Kyoto Encyclopedia of Genes and Genomes (KEGG) annotation of DEGs was carried out through the annotation tool. The analysis by Gene Ontology involves three aspects: cell components, molecular functions, and biological processes. The KEGG pathway enrichment analysis clustered DEGs into corresponding pathways for more intuitive presentation. The top 20 GO terms and top 17 KEGG terms were selected for statistical analysis, and a *P* value of less than 0.05 was set as the cutoff. The gene count arising from the GO and KEGG analyses was visually represented using Python.

### 2.5. Module Analysis of the PPIN

The Molecular Complex Detection (MCODE) (version 1.5.1) Cytoscape plugin is an application for clustering a given network based on its topology to find highly interconnected regions [21]. MCODE was used to analyze the important modules in the PPIN [22]. The parameters were set as follows: degree cutoff = 2, node density cutoff = 0.1, node score cutoff = 0.2, *K*-core = 2, and maximal depth = 100, with haircut but without loops and fluff. The TSV file of the DEG PINN was output from the STRING database and then typed into Cytoscape for module analysis. MCODE employed R language to cluster a large number of genes (proteins) into 11 core functional modules.

### 2.6. Centrality Analysis of the PPIN

In DEG PPINs, genes are abstracted as nodes or vertices while edges represent interactions between subjects. The identification of nodes is generally achieved by centrality parameter ordering. Additionally, the distribution characteristics and correlation analysis of multicentrality parameters are helpful to judge the degree of node keys and the reliability of parameters. In this study, we selected the commonly used degree, betweenness, and closeness centralities, for the investigation and prediction of key genes. Centrality parameters were calculated using the Network Analyzer Cytoscape plugin [20]. R language was then used to calculate the distribution diagram for the three key centrality parameters and correlation diagrams for each pair of the three parameters. Furthermore, the Pearson correlation coefficient was calculated to further understand the correlation of centrality parameters [21]. The intersection of the top 20% of the three centrality parameters was selected using a Venn diagram to obtain the candidate key genes.

### 2.7. Validation of mRNA Upregulation Frequency and Expression of Key Genes

With the maturation of gene chips and high-throughput sequencing technology, many genomics databases have emerged in the field of cancer research. Among these, TCGA databases are commonly used and widely recognized, which are based upon 126 sets of tumor genome research data. Some practical online analysis websites such as cBioPortal [23] (http://www.cbioportal.org/) have been derived based on TCGA. Based on multiple cancer samples, the online tool cBioPortal can calculate the frequency of changes in the expression of each candidate key gene in cancer patients.

### 2.8. Cell Culture

A normal human hepatocyte cell line (HL-7702) and HCC cell lines (SMMC-7721, MHCC-97L, and MHCC-97H) were obtained from the Chinese Academy of Sciences (Shanghai, China) [24]. HL-7702 and SMMC-7721 cells were inoculated in a 60 mm culture dish with RPMI-1640 medium containing 10% fetal bovine serum (Gibco Company, Grand Island, NY, USA) and cultured in an incubator at 37°C with 5% CO_2_ and saturated humidity. MHCC-97L and MHCC-97H cells were cultured with 90% DMEM high-glucose medium and 10% fetal bovine serum. The cell medium was replaced once every 1–2 days, and 0.25% trypsin (Sigma-Aldrich Chemical Company, St. Louis, MO, USA) was added for digestion and subculture.

### 2.9. RNA Isolation, Library Synthesis, and qRT-PCR

Total RNA was extracted from cells using the TRIzol reagent (Takara, Dalian, China) according to the manufacturer's protocols. The NanoDrop 2000 spectrophotometer (Thermo Fisher Scientific, USA) was employed to measure the OD 260/280 value of RNA specimens to enable the calculation of RNA concentration.

Reverse transcription of RNA to cDNA was performed with the PrimeScript RT reagent kit (Takara, Dalian, China) under the following conditions: 37°C for 15 min and 85°C for 5 s. Then, according to the nucleotide sequences of GAPDH, CDK1, NDC80, HMMR, CDKN3, and PTTG1 in GenBank, primers were designed by BLAST. The primer sequences are shown in Table 1. qRT-PCR was conducted using a Bio-Rad CFX96 system (Bio-Rad, CA, USA) using GAPDH as the internal reference for quantification of mRNA. A quantitative real-time fluorescence PCR reagent kit (Takara) was used to detect the messenger RNA (mRNA) expression of key genes. The reaction system (10 *μ*L) was as follows: 5 *μ*L TB Green Premix Ex Taq (Takara, Dalian, China), 0.4 *μ*L forward primer, 0.4 *μ*L reverse primer, 1 *μ*L cDNA templates, and 3.2 *μ*L ddH_2_O. The qRT-PCR conditions were as follows: predenaturation at 95°C for 3 min, 39 cycles of denaturation at 95°C for 5 s, annealing at 60°C for 30 s, extension at 72°C for 30 s, and a final elongation step at 65°C for 5 s. The relative expression of genes was calculated by the 2^–*ΔΔ*CT^ method.

### 2.10. Survival Analysis Based on Key Genes

Gene Expression Profiling Interactive Analysis (GEPIA; http://gepia.cancer-pku.cn/index.html) is a very friendly TCGA data analysis and visualization website. Based on a large volume of clinical sample data, multilevel analysis of the gene of interest can be performed. In this study, GEPIA was used to study the impact of five key genes on patient survival and prognosis.

### 2.11. Statistical Analysis

All experiments were repeated three times independently. Statistical analyses were performed using SPSS 19.0 (IBM, SPSS, Chicago, IL, USA) and GraphPad Prism 5.0 (GraphPad Software Inc., CA, USA). Data are shown as mean ± standard deviation (SD). The differences between groups were assessed by Student's *t*-test, one-way ANOVA, or the *χ*^2^ test. Survival analysis was performed using the Kaplan-Meier method and log-rank test. The Pearson correlation coefficient was used for correlation analysis. *P* < 0.05 was considered statistically significant.

## 3. Results

### 3.1. Identification of DEGs and Construction of the HCC-Related PPI Network

A total of 849 (283 upregulated and 566 downregulated) and 483 (202 upregulated and 281 downregulated) DEGs were found from GSE25097 and GSE84005, respectively, by GEO2R (∣logFC | >1.5, *q* < 0.01). Furthermore, 99 upregulated genes and 192 downregulated genes with the same expression trend in both datasets were screened out by Venny 2.1 (Figure 1(a), Table 2). The PPIN of these 291 DEGs, constructed using STRING and visualized by Cytoscape, included 287 nodes and 2527 edges (Figure 1(b)).

### 3.2. Functional Annotation of DEGs in the PPIN

To explore the functions of the DEGs in the HCC-related PPI network, GO enrichment and KEGG pathway analyses were performed using DAVID. GO enrichment showed that the genes were involved in 236 GO terms, including 52 terms relating to molecular functions, 40 terms relating to cell components, and 144 terms relating to biological processes. In these three areas, the DEGs mainly participated in the protein binding molecular function, were associated with the cytosol, and participated in the biological processes of oxidation-reduction and cell division (Figure 2(a)). Additionally, the result of KEGG pathway enrichment analysis showed that the DEGs were mainly enriched in relation to metabolism, the cell cycle, chemical carcinogenesis, P450-associated pathways, and p53 signaling pathways.

### 3.3. Module Analysis of the PPIN

To explore the significant molecules in the PPIN, module analysis was performed using Cytoscape based on files output from the STRING database. Eleven functional modules were detected (Figure 3). Specifically, the first-ranked module consisted of 61 nodes and 1704 edges, and all 61 node genes were upregulated. This suggested that the 61 molecules of the first-ranked module acted as a unit and worked together in HCC.

### 3.4. Centrality Analysis of the PPIN

To investigate the characteristics of molecules in the HCC-related PPIN, the three topological features of the network centrality—degree, betweenness, and closeness—were analyzed by the Cytoscape plugin Network Analyzer and R language. The graph shows that the degree had an atypical heavy-tailed distribution, with a peak in the tail region (Figure 4(a), left), that the betweenness had a typical heavy-tailed distribution, and the smaller the betweenness, the greater the density (Figure 4(a), middle), and that the closeness had an atypical bell-shaped distribution with double peaks (Figure 4(a), right). These results suggested that the PPIN associated with HCC was reasonable.

Additionally, the correlation between the three topological features was calculated by the R package. The analysis suggested that the degree was positively correlated with the other two centrality parameters in the HCC-related PPIN (Figure 4(b)). The Pearson coefficient of the degree and betweenness was close to 0, so the correlation between these was low (Figure 4(b), left). The Pearson coefficient of the degree and closeness was larger, indicating that they were highly correlated. The vertex with the highest score in the degree was the same high score as for the closeness (Figure 4(b), middle). The Pearson coefficient between the betweenness and the closeness was greater than 0.5, indicating that they were also highly correlated (Figure 4(b), right). These results suggested that the three topological features were important for the screening of core genes.

Furthermore, molecules in the HCC-related PPIN with topological features in the top 20% were analyzed by Venny 2.1. This revealed 10 core genes with high degree, betweenness, and closeness values, including TOP2A, CDK1, NDC80, CCNB1, HMMR, CENPF, AURKA, CDKN3, FOXM1, and PTTG1 (Figure 4(c), Table 3). Interestingly, the first-ranked module contained more than 10 core genes.

### 3.5. mRNA Upregulation Frequency and Expression of the Key Genes in HCC Cell Lines

Liver cancer samples were selected from cBioPortal (based on TCGA database) and included 429 cases of HCC, eight cases of HCC plus intrahepatic cholangiocarcinoma, three cases of fibrolamellar carcinoma, and two unconfirmed cases. The results showed five genes (CDK1, NDC80, HMMR, CDKN3, and PTTG1) that were upregulated in HCC, while the expression of the other genes varied in the different subtypes of liver cancer. Therefore, these five key genes were selected as subsequent research objects (Figure 5(a)). Additionally, to further confirm the expression of these five genes in HCC, qRT-PCR verified that the five key genes were present in a normal human liver cell line (HL-7702) and HCC cell lines (SMMC-7721, MHCC-97L, and MHCC-97H). The results showed that the expression levels of CDK1, NDC80, HMMR, CDKN3, and PTTG1 in the HCC cell lines were upregulated (Figure 5(b)). This was consistent with previous results.

### 3.6. Survival Analysis of Five Key Genes in HCC

The influence of the five key genes (CDK1, NDC80, HMMR, CDKN3, and PTTG1) on the survival of patients with HCC was analyzed using GEPIA. Results of Kaplan-Meier analysis showed that HCC patients with alterations to these five key genes had higher mortality and shorter survival periods (Figures 6(a)–6(e), Table 4). The overall survival rates of HCC patients with changes in CDK1, NDC80, HMMR, CDKN3, and PTTG1 were poor.

## 4. Discussion

HCC is the most common primary liver cancer, accounting for more than 90% of all primary liver cancers. The onset of the disease is insidious and progresses rapidly: most patients present to the hospital with terminal cancer. Although surgery, liver transplantation, radiofrequency ablation, targeted drugs, and other methods for the treatment of liver cancer have been widely used, postoperative recurrence and drug resistance are serious problems, and the prognosis is not ideal [25–27]. Recently, microarray technology, bioinformatics, and statistics have been integrated to analyze the biological behavior of HCC to achieve a new definition and classification of HCC at the molecular level.

In the present study, the two datasets GSE25097 and GSE84005 were selected from the GEO database and 291 DEGs were selected. Subsequently, an HCC-related PPIN was constructed and gene functional annotation data was analyzed. It was found that the most significant statistical pathways, according to the gene count, were the metabolic, cell cycle, and chemical carcinogenesis pathways, in that order. Among these, the cell cycle pathway is of great significance in the occurrence and development of cancer. Interestingly, many studies on HCC cell cycle pathways have shown that abnormal expression of cyclin-related genes is an important factor in the occurrence of liver cancer, and the silencing of the cyclin D1 gene inhibits the proliferation, cell cycle, and apoptosis of HCC cells [28–30]. Therefore, the present results suggested that the DEGs in the HCC-related PPIN may play an important role in the development of HCC.

Furthermore, it was found that biological function was achieved by modules made up of different molecules. MCODE analysis revealed the first-ranked module with the highest score to include 61 nodes and 1704 edges. PPIN module analysis has been widely used to identify candidate genes in various diseases. Chen et al. used PPIN module analysis to identify candidate genes for necrotizing enterocolitis based on microarray data [31]. Disease-specific PPINs are characterized by aggregation [32]. The core modules of the whole network are closely connected, while the connections between modules are sparse, indicating that the core modules were usually involved with biological functions [33]. These findings suggest that module analysis is of great significance for analyzing a PPIN.

To better explore the roles of molecules in the HCC-related PPIN, the commonly used centrality parameters—degree, betweenness, and closeness centralities—of the PPIN were calculated to determine whether the node was in an important position in the network. The centrality parameter can be used to reveal the characteristics of nodes in the network and the overall characteristics of the network [34]. The present results showed that the distributions of the degree and betweenness were characterized by heavy-tailed distribution in the PPIN, and the distribution of the closeness was bell-shaped. This indicated that only a small number of molecules interacted with most other molecules and occupied the key position of information transfer in the network. Additionally, the results of Pearson correlation analysis showed that there was a certain correlation among the centrality parameters. These results suggested that the topological characteristics of the HCC-related PPIN were obvious.

Additionally, 10 key candidate genes—TOP2A, CDK1, NDC80, CCNB1, HMMR, CENPF, AURKA, CDKN3, FOXM1, and PTTG1—were identified by the intersection of the first 20% of the three centrality parameters. Previously, Melak and Gakkhar identified drug targets of *Mycobacterium tuberculosis* H37Rv by constructing a PPIN of *Mycobacterium tuberculosis* and conducting centrality analysis [35]. Hahn and Kern found that the centrality and essentiality comparative genomics of three eukaryotic protein interaction networks, regardless of the number of direct interactors, evolved more slowly and were more likely to be essential for survival [36]. Recently, Zhang et al. identified key genes and pathways of HCC by bioinformatics and statistical methods [37]. This suggested that the 10 key candidate genes obtained through the centrality parameter analysis may be closely related to the pathogenesis of HCC. Furthermore, according to module analysis, the 10 candidate key genes with high degree, betweenness, and closeness values were all included in the first-ranked module. Therefore, these 10 candidate genes were focused on for further study.

To further investigate the influence of the 10 candidate key genes in HCC, big data validation and prognosis analysis was carried out in TCGA of large tumor databases. Results showed that CDK1, NDC80, HMMR, CDKN3, and PTTG1 were specifically upregulated in HCC. Survival analysis showed that changes in the expression of these five key genes posed a threat to the survival of patients with HCC. Furthermore, KEGG pathway correlation analysis found that they were closely related to cell cycle pathways. Additionally, these five key genes have been reported to regulate the pathogenesis of different cancers. Gan et al. found that CDK1 interacts with iASPP and can regulate the proliferation of colorectal cancer cells through the p53 pathway [38]. Elevated expression of NDC80 may play a role in promoting the development of HCC [39]. The increased expression of HMMR was associated with the progression of HCC and may be a prognostic indicator [40]. Barron et al. found that CDKN3 may be a good survival marker and potential therapeutic target for cervical cancer and that cervical cancer patients with overexpression of CDKN3 have poor survival prognosis. This suggests that CDKN3 mRNA expression levels may be a good predictor of patient survival and tumor invasiveness [41]. Romero Arenas et al. found that PTTG1 overexpression may affect the prognosis of patients with adrenal tumors and is also a promising biomarker for the evaluation of adrenal tumors [42]. Key genes CDK1, NDC80, HMMR, CDKN3, and PTTG1 have been reported to be involved in the occurrence of different cancers, suggesting that they may also play a regulatory role in the development of hepatocellular carcinoma. Additionally, cell experiments also confirmed the upregulation of CDK1, NDC80, HMMR, CDKN3, and PTTG1 in HCC. Therefore, these five key genes may be promising biomarkers for HCC, providing research directions for clinical diagnosis and prognosis analysis of HCC patients.

## 5. Conclusions

In this study, gene functional annotation analysis, module analysis, and centrality parameter analysis were conducted to search for potential HCC key genes by constructing a PPIN of DEGs. Large-sample validation analysis using TCGA database identified five key genes that were significantly enriched in the cell cycle pathway, and their expression levels and prognosis were analyzed. Additionally, differences in the expression of key genes were verified at the cell level, which needs to be further verified in HCC tissues. All these findings suggested that the five key genes may be potential targets for clinical treatment of HCC and provide further strategies for clinical diagnosis, accurate treatment, and prognosis analysis of HCC.

## Figures and Tables

**Figure 1:** Identification of DEGs and construction of the HCC-related PPI network. (a) Intersections of upregulated genes and downregulated genes from the expression profiles GSE25097 and GSE84005, as detected by Venny 2.1. (b) HCC-related PPI network, as constructed by STRING and visualized by Cytoscape. Upregulated genes are indicated with red and downregulated genes with green.

**Figure 2:** Functional annotation of DEGs. (a) GO analysis of DEGs in the HCC-related PPI network based on their molecular functions, biological processes, and cellular components. The top 20 significant terms are shown according to the gene counts (*P* < 0.05). (b) KEGG pathway analysis of DEGs in the HCC-related PPI network (*P* < 0.05).

**Figure 3:** Module analysis of the HCC-related PPI network. The network was decomposed into 11 functional modules by the Cytoscape plugin MCODE. The first-ranked module was located in the center of the PPI network and contained 61 nodes and 1704 edges.

**Figure 4:** Centrality analysis of the HCC-related PPI network. (a) Density distribution of centrality parameters (degree centrality, betweenness centrality, and closeness centrality) as calculated by the Cytoscape plugin Network Analyzer and R language. (b) Correlations among centrality parameters, as analyzed by R. (c) 10 core molecules with high degree, betweenness, and closeness centralities were selected by Venny 2.1 (top 20% of each set of centrality parameters). The first-ranked module contained 10 core molecules discovered by centrality analysis.

**Figure 5:** mRNA upregulation frequency and expression of the key genes in HCC. (a) mRNA upregulation frequency of the 10 key genes detected in primary liver cancer by cBioPortal. (b) Expression of CDK1, NDC80, HMMR, CDKN3, and PTTG1 in a normal human hepatocyte cell line (HL-7702) and HCC cell lines (SMMC-7721, MHCC-97L, and MHCC-97H) as verified by qPCR. The key genes were all upregulated in HCC cell lines. Data are shown as mean ± SD. (^∗^*P* < 0.05, ^∗∗^*P* < 0.01).

**Figure 6:** Survival analysis of the key genes in HCC by GEPIA. (a) Impact of CDK1 on the survival of HCC patients. (b) Impact of NDC80 on the survival of HCC patients. (c) Impact of HMMR on the survival of HCC patients. (d) Impact of CDKN3 on the survival of HCC patients. (e) Impact of PTTG1 on the survival of HCC patients.

**Table 1:** Primers for target genes.

Gene ID		Sequence (5′-3′)
GAPDH	Forward	GTCTTCCTGGGCAAGCAGTA
	Reverse	CTGGACAGAAACCCCACTTC
CDK1	Forward	AAGTTCAAGTTTCGTAATGC
	Reverse	ACTGTTCTTCCCTGTTGC
NDC80	Forward	TAAGTTTAATCCCGAGGCT
	Reverse	GTTGGTATTCCCGCTGA
HMMR	Forward	GCAAATACCTCCTCCCTAA
	Reverse	GGATGGAGCCTAAGAACCT
CDKN3	Forward	GGACTCCTGACATAGCCAGC
	Reverse	CTGTATTGCCCCGGATCCTC
PTTG1	Forward	ACCCGTGTGGTTGCTAAGG
	Reverse	ACGTGGTGTTGAAACTTGAGAT

**Table 2:** The 99 upregulated genes and 192 downregulated genes.

DEGs	Gene name
Upregulated genes	BUB1B, CDKN3, RACGAP1, CDCA8, MDK, KIF2C, CDCA5, GJC1, RAD51AP1, DTL, PRC1, CLGN, SKA1, COCH, PTTG1, SHCBP1, MYBL2, BRCA1, ECT2, HELLS, EXO1, ASF1B, MKI67, KIF20A, NEIL3, BUB1, FOXM1, TRIP13, SGO1, FAM83D, STIL, CENPI, CA12, MMP12, LPL, ESM1, TCF19, KIF11, GPC3, DLGAP5, MEP1A, CDK1, AURKA, depdc1b, NUSAP1, CHEK1, CCNA2, SLC7A11, CENPK, SULT1C2, KNL1, IGF2BP1, CDC20, CDC6, CCNE2, THY1, E2F8, CCNB2, TOP2A, MUC13, SKA3, ASPM, FANCI, TTC39A, CCNB1, NCAPG, SPINK1, CD109, SPDL1, MCM8, FLVCR1, KIF14, GNG4, NUF2, KIF4A, DNAJC6, RRM2, MELK, ANLN, PBK, NCAPH, UBE2T, HMMR, SQLE, FAM111B, EZH2, CKAP2, AKR1B10, TTK, CDC25C, ATAD2, MCM2, KIF23, NQO1, SPC25, TPX2, HJURP, CENPF, NDC80
Downregulated genes	LUM, DCN, RANBP3L, NNMT, timd4, CLEC1B, PTPRB, HPD, OAT, PLAC8, CYP3A43, ADRA1A, KCNN2, FBLN5, HGFAC, MS4A6A, CXCL12, SFRP5, HAMP, CTH, MBL2, EPHA3, MFSD2A, IYD, MASP2, LY6E, CDHR2, CD163, AKR1D1, SRPX, GZMK, SHBG, ACADL, FAM180A, LCAT, FREM2, VIPR1, Ugt2b10, SLC10A1, AADAT, SLC4A4, CHST4, MT1G, C9, ABCA8, ADGRE1, ADGRG7, HAO2, NAT2, BBOX1, FCN3, PAMR1, ALPL, SLC16A4, fam134b, UGT2B7, LIFR, PROZ, CPED1, CETP, ID1, DNASE1L3, GPD1, GPM6A, RDH16, FCN2, rspo3, EHD3, TEK, PRKAR2B, GYS2, RND3, IGF1, FOSB, BCHE, SDS, RDH5, C6, TMEM27, SPP2, FXYD1, GLS2, ENO3, FOS, GNMT, MT1X, MME, ABCA9, RELN, RAB25, LAMA2, ADH4, GBA3, APOF, CYP1A1, Mt1m, NPY1R, IL7R, SLC1A2, CYP39A1, CFTR, MT1A, Mt1f, DPT, COLEC11, CYP26A1, SLC25A47, THRSP, UROC1, TFPI2, CCL21, BMP5, STAB2, BCO2, CCDC3, Cyp1a2, APOA5, MFAP4, HAND2-AS1, CYP2E1, CYP2C8, CYP2C9, CYP4A11, SLC22A1, GLYAT, COLEC10, INMT, CFHR3, MARCO, ECM1, BMPER, CRHBP, MT1P3, LRAT, LOC100287413, MT1L, SELP, HGF, MFAP3L, TDO2, CLEC4G, GNA14, SLCO1B3, SPIC, SCIMP, HSD17B13, CCBE1, LPA, cyp3a4, clrn3, KMO, CYP8B1, OGDHL, acsm3, RBMS3, SULT1E1, OIT3, SULT1B1, CD69, DNAJC12, XDH, MMRN1, STEAP4, CNDP1, IL13RA2, CD5L, c8orf4, SRD5A2, ASPN, SLC5A1, GHR, CFP, SLC22A10, ITGA9, C7, HSD11B1, CCL19, S100A8, AFM, LYVE1, P2RY13, HHIP, JCHAIN, RBP1, CXCL2, PZP, cyp2c19, IDO2, CLEC12A, DIRAS3, CXCL14, ANGPTL1

**Table 3:** Ten key molecules with high centralities in the PPI network.

Gene name	Description	Degree	Betweenness	Closeness
TOP2A	DNA topoisomerase II alpha	93	0.29654147	0.4845815
CDK1	Cyclin-dependent kinase 1	74	0.01937521	0.43737575
NDC80	NDC80 kinetochore complex component	73	0.06677326	0.44088176
CCNB1	Cyclin B1	73	0.01896303	0.43650794
HMMR	Hyaluronan-mediated motility receptor	71	0.03418334	0.4206501
CENPF	Centromere protein F	70	0.03351845	0.43222004
AURKA	Aurora kinase A	69	0.02444692	0.4238921
CDKN3	Cyclin-dependent kinase inhibitor 3	67	0.02961628	0.43650794
FOXM1	Forkhead box M1	62	0.06382427	0.44534413
PTTG1	PTTG1 regulator of sister chromatid separation, securin	60	0.01557241	0.4206501

**Table 4:** The aliases and gene function of 5 key genes.

Gene symbol	Aliases	Gene function
CDK1	CDC2, CDC28A, P34CDC2	This gene is essential for G1/S and G2/M phase transitions of the eukaryotic cell cycle.
NDC80	HEC, HEC1, TID3, KNTC2, HsHec1, hsNDC80	The gene encodes proteins necessary for proper chromosome segregation.
HMMR	CD168, IHABP, RHAMM	The protein encoded by this gene is involved in cell motility and potentially associated with a higher risk of breast cancer.
CDKN3	CDKN3, CDI1, CIP2, KAP	The protein encoded by this gene belongs to the dual-specificity protein phosphatase family. This gene was reported to be deleted, mutated, or overexpressed in several kinds of cancers.
PTTG1	EAP1, HPTTG, MGC126883, MGC138276, PTTG, TUTR1	The gene product contains 2 PXXP motifs, which are required for its transforming and tumorigenic activities, as well as for its stimulation of basic fibroblast growth factor expression.

## Data Availability

Some or all data, models, or codes generated or used during the study are available from the corresponding author by request.
